RETRACTED

# BRD7 inhibits the Warburg effect and tumor progression through inactivation of HIF1α/LDHA axis in breast cancer

**DOI:** 10.1038/s41419-018-0536-7

**Published:** 2018-05-03

**Authors:** Weihong Niu, Yanwei Luo, Xinye Wang, Yao Zhou, Hui Li, Heran Wang, Yaojie Fu, Shanshan Liu, Shanghelin Yin, Jianglei Li, Ran Zhao, Yukun Liu, Songqing Fan, Zheng Li, Wei Xiong, Xiaoling Li, Guiyuan Li, Caiping Ren, Ming Tan, Ming Zhou

**Affiliations:** 1 The Affiliated Tumor Hospital of Xiangya Medical School, Central South University, Changsha, Hunan 410013 People’s Republic of China; 2 The Key Laboratory of Carcinogenesis of the Chinese Ministry of Health, The Key Laboratory of Carcinogenesis and Cancer Invasion of the Chinese Ministry of Education, Xiangya Hospital, Central South University, Changsha, Hunan 410078 People’s Republic of China; 3 Cancer Research Institute, Central South University, Changsha, Hunan 410078 People’s Republic of China; 4 The Second Xiang-Ya Hospital, Central South University, Changsha, Hunan 410011 People’s Republic of China; 5 Medical school of Xiangya, Central South University, Changsha, Hunan 410013 People’s Republic of China; 6 High Resolution Mass Spectrometry Laboratory of Advanced Research Center, Central South University, Changsha, Hunan 410013 People’s Republic of China; 7 Mitchell Cancer Institute, University of South Alabama, Mobile, AL 36604 USA

## Abstract

The bromodomain-containing protein 7 (BRD7) was first identified as a tumor suppressor in nasopharyngeal carcinoma and has critical roles in cancer development and progression. However, the regulatory roles and mechanisms of BRD7 in cancer metabolism are still unknown. In this study, we demonstrated that BRD7 was lowly expressed in breast cancer tissues and was identified as a poor prognostic factor in breast cancer. Meanwhile, BRD7 could suppress cell proliferation, initiate cell apoptosis and reduce aerobic glycolysis, suggesting that BRD7 plays a tumor suppressive roles in breast cancer. Mechanistically, BRD7 could negatively regulate a critical glycolytic enzyme LDHA through directly interaction with its upstream transcription factor, HIF1α, facilitating degradation of HIF1α mediated by ubiquitin–proteasome pathway. Moreover, restoring the expression of LDHA in breast cancer cells could reverse the effect of BRD7 on aerobic glycolysis, cell proliferation, and tumor formation, as well as the expression of cell cycle and apopotosis related molecules such as cyclin D1, CDK4, P21, and c-PARP both in vitro and in vivo. Taken together, these results indicate that BRD7 acts as a tumor suppressor in breast cancer and represses the glycolysis and tumor progression through inactivation of HIF1α/LDHA transcription axis.

RETRACTED

## Introduction

Bromodomain-containing proteins are a class of evolutionarily conserved proteins that includes bromodomain-containing protein 7 (BRD7). Since our group first cloned this gene from nasopharyngeal carcinoma (NPC) cells in 2000, numerous studies have shown that BRD7 plays critical roles in cancer development and progression^1–3^. Our previous studies have demonstrated that BRD7 is involved in growth inhibition of NPC by inhibiting cell cycle progression from G1 to S, and thus was identified as a tumor suppressor in NPC^4,5^. BRD7 is also involved in multiple physiological processes, including the regulation of spermatogenesis and cognitive behavior^6–8^. BRD7 is downregulated in multiple types of tumor specimen and cancer cells, and might be involved in the development and progression of multiple types of cancers, including breast cancer and prostate cancer^1^. BRD7 can bind to BRCA1 in breast cancer cells, which is required for the BRCA1-mediated transcriptional regulation of the estrogen receptor (ER), suggesting a close relationship between BRD7 and breast cancer development^9^. However, so far there is still no direct evidence to show that BRD7 plays a role in breast cancer.

Interaction of BRD7 and p53 is essential for the transcriptional activation of some target genes of p53, including p21 and MDM2, which is required for p53-dependent oncogene-induced senescence^10,11^. Notably, one study shows that BRD7 is capable of regulating X-box binding protein 1 (XBP1) nuclear translocation and interacts with the regulatory subunits of phosphatidyl-inositol3-kinase (PI3K) to increase the nuclear translocation of both p85α/β and XBP1s. Reinstating BRD7 levels in the liver restores XBP1s nuclear translocation, improves glucose homeostasis^12^, and ultimately reduces the blood glucose levels in obese and diabetic mouse models^13^, which is also consistent with the result of the recent paper, the role of BRD7 in embryo development and glucose metabolism, suggesting that BRD7 is implicated in cellular energy metabolism mechanisms such as glycolysis. However, the role of BRD7 in regulating cancer cell metabolism has not been systematically investigated. Hypoxia-inducible factor 1α (HIF1α) takes part in the reprogramming of cancer metabolism by regulating key molecules, including LDHA, SLC2A1, SLC2A3, HK1, HK2, and MCT4 in glucose metabolism^14,15^. The expression of HIF1α is high in multiple types of cancers, such as lung cancer, prostate cancer, breast cancer, and colonic adenocarcinoma. In tumor progression, insulin, insulin-like growth factor (IGF)-1 or IGF-2, v-Src, lactate, pyruvate, and genetic alterations such as oncogene activation or tumor suppressor gene inactivation lead to HIF1α overexpression^14,16^.

RETRACTED

Mounting evidence accumulated in cancer research has demonstrated that dysregulated cancer cell bioenergy plays an important role in the development and progression of breast cancer^17^. While currently there is no direct evidence to support a role of BRD7 in breast cancer and it is not clear whether BRD7 regulates cancer cell metabolism. Therefore, in this study we investigated whether BRD7 indeed plays a role in breast cancer progression and explored whether BRD7 regulates breast cancer cell metabolism. We revealed that BRD7 showed low expression in breast cancer tissues compared to normal tissue, and loss of BRD7 expression in breast cancer was identified as a poor prognostic factor. Moreover, ectopic expression of BRD7 in breast cancer cells suppressed cell proliferation, initiated cell apoptosis, and decreased glycolysis. Furthermore, we found that lactate dehydrogenase A (LDHA) was negatively regulated by BRD7 through promoting proteasomal degradation of HIF1α, and restoring the expression of LDHA in BRD7-overexpressed or breast cancer cells could reverse the effect of BRD7 on aerobic glycolysis, cell proliferation, and apoptosis, as well as the expression of cell cycle and apopotosis related molecules such as cyclin D1, CDK4, P21, and c-poly-ADP-ribose polymerase (c-PARP) both in vitro and in vivo. Taken together, these results indicate that BRD7 functions as a tumor suppressor gene in breast cancer and BRD7 inhibits aerobic glycolysis and tumor progression through inactivation of HIF1α/LDHA transcription axis.

## Materials and Methods

### Tissue samples and clinical data

All the human tissues were collected from the Second Xiangya Hospital of Central South University from November 2001 to September 2012. This study was approved by the Committee on the Ethics of Central South University. All of the individuals participating in this study have provided written informed consent. The samples were compiled into a tissue microarray as previously described, which included 225 cases of breast cancer tissues and 61 cases of non-cancerous breast tissues^18–20^. Clinicopathologic characteristics of breast cancer patients were recorded, including gender, age, clinical tumor node metastasis (TNM) stage, pathology diagnosis, and molecular subtype. The profile of clinicopathologic characteristics of the breast cancer patients is shown in Table 1. Patients’ ages ranged from 23 to 71 years old. All of the 225 breast cancer patients had valid follow-up data, and the longest survival time was 120 months. The overall survival (OS) was defined as the time from diagnosis to the date of death or the date last known alive.

RETRACTED

**Table 1:** Clinicopathologic characteristics of breast cancer patients

Age	
Mean ± S.D.	46 ± 0.66
Sex (%)	
Male	0.4 (1/225)
Female	99.6 (224/225)
Tumor size (%)	
T1–2	62.7 (141/225)
T3–4	37.3 (84/225)
Nodal metastasis (%)	
Present	74.2 (167/225)
Absent	25.8 (58/225)
Distant metastasis (%)	
Present	9.3 (21/225)
Absent	81.7 (204/225)
TNM stage (%)	
I–II	65.8 (148/225)
III–IV	34.2 (77/225)

### Cell culture

Human breast cancer cell lines MCF-7, MDA-MB-231, MDA-MB-453, and the human embryonic kidney cell line HEK-293T were obtained from the American Type Culture Collection (Manassas, VA, USA). All cells were cultured in high glucose DMEM medium (Invitrogen Life Technologies, Carlsbad, CA, USA) containing 10% fetal bovine serum (FBS) (Gibco, Thermo Fisher Scientific, Waltham, MA, USA), 100 units/ml penicillin and 100 mg/ml streptomycin. The cells were incubated at 37 °C in 5% CO_2_. For hypoxic condition, cells were cultured in a Hypoxic Workstation (Don Whitley, West Yorkshire, UK) that was infused with a mixture of 1% O_2_, 5% CO_2_ and at 37 °C temperature. Cells were lysed for extraction of protein and RNA in the workstation to avoid reoxygenation.

### Transfection

For ectopic expression of BRD7 in MCF-7, MDA-MB-231, and MDA-MB-453, the cells were transfected with pIRES2-EGFP-3Flag/BRD7 using Lipofectamine 3000 transfection reagent (Invitrogen, Carlsbad, CA) according to the manufacturer’s instructions; the cells transfected with pIRES2-EGFP were used as a negative control. The positive cells with ectopic expression of BRD7 or blank control were further sorted by GFP-mediated flow cytometry technology and extended culture. As for the recovery experiment for LDHA, the MCF-7, MDA-MB-231, and MDA-MB-453 cells with BRD7 overexpression were further transiently transfected with pENTER/LDHA or pENTER, and the cells transfected with pIRES2-EGFP and pENTER vectors were used as a control. To knock down BRD7 or LDHA expression in MCF-7 and MDA-MB-231 cells, the cells were transfected with BRD7 or LDHA small interfering RNA (siRNA) oligonucleotides (Ribobio, Guang zhou; 50 nmol/l). The cells transfected with control siRNA oligonucleotides were used as a negative control.

### Inhibition of glycolysis with oxamate and 2-DG

To inhibit aerobic glycolysis in breast cancer cells, the glycolytic inhibitors oxamate sodium (Oxamate; Sigma-Aldrich, St. Louis, MO, USA) and 2-deoxy-d-glucose (2-DG) (Sigma-Aldrich, St. Louis, MO, USA) were used to treat the breast cancer cells (MCF-7 and MDA-MD-231) with ectopic expression of BRD7 sorted by GFP-mediated flow cytometry technology at different concentrations. For oxamate, the cells were treated with a concentration of 50 or 80 mM for different lengths of time (48 or 72 h). For 2-DG, the cells were treated with various concentrations (2, 4, 6 mM) of 2-DG for 48 h. Then, the cell viability was measured using an MTT assay, and the data were presented as the percentage of viability inhibition.

RETRACTED

### Immunohistochemistry

The paraffin-embedded slides were routinely deparaffinized and hydrated. The slides were then retrieved in citric acid buffer (pH 6.0), heated in a microwave oven for 10 min, and then treated with 3% H_2_O_2_ for 15 min and washed with Tris-buffered saline containing 1% Tween 20 (TBST) three times each for 5 min. After a 60 min incubation in normal goat serum (Boster, Wuhan, China), the slides were incubated with primary antibodies overnight at 4°C. The antibodies included polyclonal rabbit anti-BRD7 (1:500 dilution), polyclonal rabbit anti-LDHA (1:2000 dilution) from Proteintech (Wuhan, China), polyclonal rabbit polyclonal rabbit anti-Cyclin D1 (1:200 dilution) from Santa Cruz (Dallas, TX, USA), polyclonal rabbit anti-c-PARP (1:200 dilution) and polyclonal rabbit anti-p21 (1:500 dilution) from Cell Signaling Technology (Danvers, MA), and polyclonal rabbit anti-Ki67 (1:200 dilution) from Bioworld Technology, Inc. (St. Louis, Minnesota, USA). The slides were washed three times with TBST (each for 15 min) and then incubated with a secondary goat anti-rabbit antibody (Maixin, Fujian, China) for 60 min at 37 °C. Then, the slides were visualized with 3,3′-diaminobenzidine (DAB) (Zhongshan Gold Bridge, Beijing, China) for 5 min and counterstained with hematoxylin for 45 s. The slides were mounted and photographed with an Olympus BX51 microscope (Olympus, Japan).

### Evaluation of staining

To evaluate the expression of BRD7 in the tissue microarrays, two independent pathologists who blinded to clinicopathologic features and clinical scored the staining under a light microscope (BX51; Olympus, Japan). BRD7 staining intensity was scored as 0 (negative, −), 1 (weak, +), 2 (moderate, ++), and 3 (strong, +++). The extent of staining was scored as 0–1.0 (0–100%). The final staining score (0–3) was calculated as the multiplication of the intensity score and extent score. The value of final score ≥1 was defined as high expression, otherwise was defined as low expression, which was referred to the previous publication^18,19^.

To semi-quantify the expression of BRD7, LDHA, Cyclin D1, p21, c-PARP, and Ki67 in the tumor tissues from nude mice, Image-J (NIH) was used to access the integral optical density (IOD) of immunoreactivity. Data were acquired from eight sections/animal and averaged to produce a single value per subject.

RETRACTED

### Immunoprecipitation

After transfection, MCF-7 cells were cultured in a hypoxic workstation with 1% O_2_ for 24 h. Then the media covering the cells were washed once with phosphate-buffered saline (PBS). Cells were then scraped from the plates in 500 μl of ice-cold RIPA lysis buffer containing protease and phosphatase inhibitors (Roche). The lysed cells were pipetted into a 1.5 ml Eppendorf tube, incubated on ice for 30 min, and microcentrifuged at 13,000 rpm for 15 min at 4 °C. Clarified lysates were incubated with 2 μg indicated antibody overnight at 4 °C, and then incubated for 2 h with 30 μl Protein A/G Agarose. Beads were extensively washed in lysis buffer, and bound proteins were eluted in moderate 2× SDS sample buffer for 100 °C 10 min and subjected to western blot analysis.

### Ubiquitination assay

MCF-7 cells were transiently transfected with the indicated plasmids and treated with MG132 (10 µM) for 8 h prior to cell lysis and in a hypoxic workstation with 1% O_2_ for 24 h. Subsequently, cells were washed with ice-cold PBS and lysed in ice-cold RIPA lysis buffer containing protease and phosphatase inhibitors. Next, cell lysates were cleared by a spin (13,000 rpm, 15 min, 4 °C) and a fixed amount of whole-cell lysates was incubated with the HIF1α antibodies (1:1000 dilution) from Abcam (Cambridge, MA) overnight. Then bound proteins were eluted in moderate 2× SDS sample buffer at 100 °C for 10 min and subjected to western blot analysis.

### Protein stability and half-life assay

MCF-7 cells were transiently transfected with the indicated plasmids. Twenty-four hours later, the cells were treated with 10 µM MG132 (Selleckchem, Houston, USA) and 150 μM CoCl_2_ (Sigma-Aldrich, St. Louis, MO, USA) prior to cell lysis for indicated time (0, 4, 8, 12, 16 h). To test the half-life of HIF1α, the transfected MCF-7 cells were firstly treated with 150 μM CoCl_2_ for 24 h, then the cells were incubated with 50 μg/ml cycloheximide (CHX; MedChemExpress, USA), a kind of protein synthesis inhibitor, for the indicated periods of time (0, 1, 3, 6 h). Finally, the above whole-cell lysate was subjected to western blot analysis.

### Western blot

Protein was extracted from indicated cells by using RIPA lysis buffer. Protein concentrations were determined using a BCA Protein Assay kit (Thermo Fisher Scientific, Rockford, IL, USA). A total of 60 μg of protein was separated on a 10% SDS-PAGE gel and transferred onto polyvinylidene difluoride membranes (Millipore, Billerica, MA, USA), which were soaked in 5% nonfat milk for 1 h and then incubated with corresponding primary antibodies overnight at 4 °C. Antibodies used in this study: rabbit polyclonal anti-BRD7 (1:500 dilution), rabbit polyclonal anti-LDHA (1:20,000 dilution), and rabbit polyclonal anti-β-Tubulin (1:3000 dilution) from Proteintech (Wuhan, China); rabbit polyclonal anti-t-PARP (1:1000 dilution), rabbit polyclonal anti-c-PARP (1:500 dilution), and rabbit polyclonal anti-p21 (1:1000 dilution) from Cell Signaling Technology (Danvers, MA); rabbit polyclonal anti-Cyclin D1 (1:500 dilution), rabbit polyclonal anti-CDK4 (1:500 dilution), and rabbit polyclonal anti-UB (1:3000 dilution) from Santa Cruz (Dallas, Texas, USA); mouse monoclonal anti-HIF1α (1:1000 dilution) from Abcam (Cambridge, USA). After washing with 1× TBST three times for 8 min each, the membranes were incubated with the corresponding secondary antibodies for 1 h at 37 °C, and then washed with 1× TBST for three times again, and finally the bands were visualized using an ECL kit (Millipore). Signals were quantified by Image-J software and normalized to β-tubulin.

RETRACTED

### Lactate production assay and LDH activity assay

Cells were seeded on six-well plates at a density of 1 × 10^5^ cells per well, and the culture medium was changed to fresh DMEM medium after incubation overnight. Lactate concentrations in the culture medium were collected and measured after 24 or 48 h using a Lactate Assay Kit (Jiancheng Bioengineering, Nanjing, China). Meanwhile, the cells were lysed in isolation buffer provided in the LDH activity assay kit (Jiancheng Bioengineering, Nanjing, China), and the LDH activity was determined according to the manufacturer’s instructions. Total enzyme activity was normalized to the protein content of the cell lysate.

### Measurement of ATP content and pyruvate dehydrogenase activity

The ATP concentration was measured by a firefly luciferase-based Bioluminescence ATP assay kit (Beyotime Biotechnology) following the manufacturer’s protocol^21^. For immune-captured pyruvate dehydrogenase (PDH) activity, the pyruvate dehydrogenase Elisa assay (Jiancheng Bioengineering, Nanjing, China) was used according to the manufacturer’s instructions^22^. The PDH activity and ATP concentration detected by using a PARADIGM Detection Platform (Beckman, Brea, CA). Values were normalized to the protein content of the cell lysate and expressed as a fold increase over vector control.

### Cell viability measurement

One thousand cells were seeded into each well of a 96-well plate and cultured for 0, 24, 48, 72, and 96 h continuously. At each time point, 200 μl of MTT (Sigma-Aldrich, St. Louis, MO, USA) at a 0.5 mg/ml final concentration was added into each well and incubated for 4 h at 37 °C. Then 150 μl of DMSO (Sigma-Aldrich) was added to each well and incubated for 10 min at room temperature. Finally, the optical density (OD) at 490 nm was detected by using a PARADIGM Detection Platform (Beckman, Brea, CA). The experiments were repeated three independent times.

RETRACTED

### Colony formation assay

A total of three hundred cells in each group were added to each well of a six-well plate in triplicate for 10–12 days. Then, the colonies were fixed and stained with crystal violet. The colony number was counted in each group. Each experiment had three duplicates and was conducted independently.

### Cell cycle analysis

Cells from each group were washed with cold PBS and collected. The cells were fixed in 70% alcohol at 4 °C overnight. Then, the cells were treated with RNase A (TaKaRa, Japan) for 30 min at 37 °C and stained with propidium iodide (PI) (KeyGEN Biotech) for 15 min, protected from light. The cell cycle was analyzed by using BD LSRFortessa (Becton, Dickinson and Company) and Mod fit LT software (Verity Software House, Topsham, ME). This assay was repeated three independent times.

### Cell apoptosis assay

An Annexin V-PE/7-AAD Apoptosis Detection Kit (BD, Biosciences) was used to detect cell apoptosis. After the indicated treatment, the cells were collected and washed twice with cold PBS and then resuspended in 100 μl of 1× binding buffer. A volume of 5 μl of Annexin V-PE and 5 μl of 7-AAD was added, mixed well, and incubated for 10 min, protected from light. Cells were analyzed using BD LSRFortessa (Becton, Dickinson and Company, Franklin Lakes, New Jersey, USA). This assay was repeated three independent times.

### Luciferase reporter gene assays

A 1.8 kb LDHA promoter sequence from −1683 to +138 bp relative to the transcription initiation site was inserted into the pGL3-echancer vector (Promega) to generate a recombinant luciferase reporter gene (pluc-LDHA). HEK293, MCF-7, and MDA-MB-231 cells were transfected with the pLuc-LDHA alone or co-transfected with a BRD7 expressed plasmid or vector control. The cells transfected with empty pGL3-echancer vector were used as a control. At 36 h after transfection, cells were collected and lysed. A volume of 100 μl of the supernatants was used to detect luciferase activities using a luciferase reporter gene assay kit (Promega, Madison, WI, USA) on the PARADIGM Detection Platform (Beckman, Brea, CA).

### Chromatin immunoprecipitation assay

MCF-7 cells were crosslinked in 1% formaldehyde for 10 min at 37 °C. DNA from fixed chromatin cells was then subjected to immunoprecipitation using a ChIP assay kit (Millipore) and antibodies against Flag (Sigma-Aldrich, St. Louis, MO, USA) or anti-mouse IgG (Santa Cruz, Dallas) according to the manufacturer’s protocol. On the basis of the requirement of the ChIP assay, the 1.8-kb promoter region of LDHA was divided into nine fragments based on the DNA walking method. Each of the fragments was approximately 200–240 bp length. The primers of each fragments are as follows: P1: 5′-TGGCCCACCCCTAAACTTTC-3′ (Forward), 5′-ACTCATGCCTGTAATCCCAGCA-3′ (Reverse); P2: 5′-GCTGGGATTCAGGC ATGAGT-3′ (Forward), 5′-AGATAGCCTCAGGAAGGAGC-3′ (Reverse); P3: 5′- GCTCCTTCCTGAGGCTATCTA-3′ (Forward), 5′-ACCTCTGGGCCTGTATTCT T-3′ (Reverse); P4: 5′**-**CAAGAATACAGGCCCAGAGG-3′ (Forward), 5′-CCTGCC TCAGCCTCCTGAG-3′ (Reverse); P5: 5′-TTCTCAGGAG GCTGAGGCAG-3′ (Forward), 5′-ATGGCTTCCTGCAGCCTCG-3′ (Reverse); P6: 5′-GCTTGTAGT CCCAGTCACTTCG-3′ (Forward), 5′-ACCCCACTGGCATCTCATCTC-3′ (Reverse); P7: 5′-CTGACAGTTCTTGGGTATGGTTG-3′ (Forward), 5′-GAAG AAAATGCCTAGCAT CAGTC-3′ (Reverse); P8: 5′-CTGACTGCTAGGCATTTTC TTC-3′ (Forward), 5′-CAACCACA GAAGCCGGGGT-3′ (Reverse); P9: 5′-ACT CAGGCTCATGGCTCCG-3′ (Forward), 5′-AGCTATGCTGACGTCAGCGG-3′ (Reverse). The primer pair from the binding region of BIRC2, 5′-CACAGTGG TTGCTGTCAAGG-3′ (Forward) and 5′-CTGGCCCTTTAACCCTGTCT-3′ (Reverse) was used as a positive control^5^. The PCR products were resolved electrophoretically on a 1.5% agarose gel and visualized using ethidium bromide staining.

RETRACTED

### Immunofluorescence staining

For detection of co-localization of BRD7 and HIF1α, after fixation with 4% paraformaldehyde and permeabilization in 0.3% TritonX-100, cells were incubated with the indicated BRD7 and HIF1α antibodies (1:200 dilution) for 16 h at 4 °C. The samples were immunostained with Alexa Fluor 488-conjugated anti-rabbit IgG polyclonal (1:1000 dilution) and Alexa Fluor 594-conjugated anti-mouse IgG (1:1000 dilution) from Life Technology (Carlsbad, CA, USA), for 1 h at 37 °C. Then cells were incubated with 4′,6-diamidino-2-phenylindole (DAPI; 1:1000 dilution) for 10 min at room temperature. Images were collected using a confocal fluorescence microscope from UltraView Vox, PerkinElmer, USA.

### In vivo tumorigenicity assays

Xenograft tumorigenicity assays were approved by the Institutional Animal Care and Use Committee of Central South University (Changsha, China). Five-week-old female athymic nude mice were divided into three groups, each group containing five female athymic nude mice. Mice were injected intramuscularly with 0.2 mg of 17-β-estradiol in 10 μl of ethyl alcohol (Tokyo Chemical Industry, Tokyo, Japan) every 2 days for 6 days before injection of MCF-7 cells. The three groups of MCF-7 cells were prepared as described in the above in intro experiments, including MCF-7 cells transfected with pIRES2-EGFP-3Flag/BRD7 alone, co-transfected with pIRES2-EGFP-3Flag/BRD7 and pENTER/LDHA, and the cells transfected with pIRES2-EGFP and pENTER were used as a control. After the indicated treatment, 5 × 10^6^ MCF-7 cells in 150 μl of normal saline were injected subcutaneously into the subaxillary of the right forelimb. Mice were examined, and tumor volumes were measured every 2 days. Twenty days after injection, all mice were sacrificed to examine the final tumor weight and the expression of key molecules related to cell cycle and apoptosis. The tumor volume was equivalent to 1/2 (length × width^2^). Tumor weight was also recorded when mice executed. All animals were allowed access to standard chow diet and water ad libitum and were housed in a pathogen-free barrier facility with a 12 L:12D cycle. The mice were sacrificed by CO_2_ asphyxiation.

RETRACTED

### Statistical analysis

GraphPad Prism 6 software (Graphpad Software, Inc., La Jolla, CA, USA) and SPSS 18.0 were used to perform statistical analysis. The data were presented as the mean ± standard deviation. The contingency data were analyzed using the chi-squared test. The OS estimates over time were calculated using the Kaplan–Meier method with log-rank test. Student’s *t*-test and ANOVA were used depending on experimental conditions. A value of *P* < 0.05 was considered to be statistically significant.

## Results

### Low expression of BRD7 predicts a poor prognosis in patients with breast cancer

We detected the expression of BRD7 in breast cancer and non-cancerous breast tissues by immunohistochemistry and the clinicopathologic characteristics of breast cancer patients are shown in Table 1. As a result, BRD7 was diffusely expressed in the cytoplasm and nucleus of breast cancer cells but mainly expressed in the nucleus (Fig. 1a). The average expression of BRD7 in breast cancer tissues was lower than that in the non-cancerous breast control tissues (Fig. 1b), and the percentage of high BRD7 expression in the breast cancer and the non-cancerous breast tissue was 58.7% (132/225) and 83.6% (51/61), respectively. In addition, the expression of BRD7 decreased with an increase in the clinical TNM stage of breast cancer patients (Fig. 1a, c and Table 2).

**Fig. 1:** BRD7 expression was negatively correlated with clinical stage and poor prognosis in breast cancer. **a** Representative images of immunohistochemistry staining for BRD7 in non-cancerous breast tissues and different clinical TNM stage I–IV breast cancer tissues. Upper bar = 200 μm; lower bar = 50 μm. **b** The score of BRD7 expression in normal adjacent tissues and breast cancer tissues. **c** The relative BRD7 expression in normal adjacent tissues and different clinical TNM stages of breast cancer tissues. **d** Kaplan–Meier curves showed worse overall survival rates for breast cancer patients with low expression of BRD7 compared to patients with high expression of BRD7 (*P* = 0.0004). Data are expressed as the mean ± S.D. *P < 0.05, **P < 0.01, ***P < 0.001

**Table 2:** Association between BRD7 expression and clinicopathologic characteristics in breast cancer

Variables	BRD7 expression		*χ*^2^ test P
	High (score≥1), *n*=132	Low (score<1), *n*=93	
Age	46.13 ± 0.92 (58.7)	46.73 ± 0.94 (41.3)	0.65
Sex (%)			1.00
Male	1 (0.7)	0 (0)	
Female	131 (99.3)	93 (100)	
Tumor size (%)			0.025*
T1–2	91 (68.9)	50 (53.7)	
T3–4	41 (31.1)	43 (46.2)	
Nodal metastasis (%)			0.87
Present	97 (73.5)	70 (75.3)	
Absent	35 (26.5)	23 (24.7)	
Distant metastasis (%)			0.061
Present	8 (6.1)	13 (14.0)	
Absent	124 (93.9)	80 (86.0)	
TNM stage (%)			0.002**
I–II	98 (74.2)	50 (53.8)	
III–IV	34 (25.8)	43 (46.2)	
ER expression (%)			0.021*
Positive	78 (59.1)	40 (43.0)	
Negative	54 (40.9)	53 (57.0)	
PR expression (%)			0.227
Positive	72 (54.5)	43 (46.2)	
Negative	60 (45.5)	50 (53.8)	
HER2 expression (%)			0.039*
Positive	71 (53.8)	63 (67.7)	
Negative	61 (46.2)	30 (32.3)	

*TNM* Tumor Node Metastasis, *ER* estrogen receptors, *PR* progesterone receptors, *HER* human epidermal growth factor receptor-2, *P* pathological. ^*^P < 0.05, **P < 0.01

We further investigated the association between the expression of the BRD7 protein and clinicopathological features of breast cancer. As shown in Table 2, no significant differences were observed between BRD7 protein expression and age, gender, lymph node metastasis, or PR expression of breast cancer (*P* > 0.05). However, BRD7 expression was significantly associated with the tumor size (*P* = 0.025), clinical TNM stage (*P* = 0.002), ER expression (*P* = 0.02), and HER2 expression (*P* = 0.039). We also analyzed the association between BRD7 expression and survival of the patients. All 225 breast cancer patients were included in the survival curves. The survival time ranged from 2 to 120 months. The OS rate of patients with high BRD7 expression is significantly higher than the survival of patients with low BRD7 expression (*P* = 0.0004, Hazard ratio = 2.83, 95% CI of ratio: 1.59 to 5.05, Fig. 1d). These results indicate that BRD7 has an essential role in the development of breast cancer.

RETRACTED

### Ectopic expression of BRD7 inhibits cell proliferation and induces apoptosis

To further investigate the tumor suppressive role of BRD7 in breast cancer, we firstly detected the expression of exogenous BRD7 and the effect of ectopic expression of BRD7 on cell proliferation and apoptosis in breast cancer MCF-7 and MDA-MB-231 cells. The result showed a significant increase in BRD7 expression compared with the control group (Fig. 2a). As we expected, overexpression of BRD7 significantly inhibited cell proliferation and colony formation (Fig. 2b, c), arrested cell cycle progression at the G1/S phase (Fig. 2d), and initiated apoptosis (Fig. 2e) in both MCF-7 and MDA-MB-231 cell lines. As BRD7 is correlated with HER2 (Table 2), while both of MCF-7 and MDA-MB-231 are HER2-negative cells, we chose another HER2-positive MDA-MB-453 cell line to repeat our results. As a result, ectopic expression of BRD7 significantly inhibited cell proliferation, arrested cell cycle progression at the G1/S phase, and initiated apoptosis (Supplementary Fig. 2a–c) in MDA-MB-453 cells, which is consistent with the results shown in HER2-negative breast cancer cells. Altogether, these results indicate that BRD7 functions as a tumor suppressor whether in HER2-negative or positive breast cancer cells.

**Fig. 2:** BRD7 inhibits cell proliferation and induces cell apoptosis in breast cancer cells. **a** Western blot analysis of the expression of BRD7 in MCF-7 (left) and MDA-MB-231 (right) cells transfected with pIRES2-EGFP-3Flag/BRD7. **b** MTT assay in MCF-7 and MDA-MB-231 cells transfected with pIRES2-EGFP-3Flag/BRD7 or pIRES2-EGFP. **c** Colony formation assay was used to determine the colony forming ability in MCF-7 and MDA-MB-231 cells transfected with pIRES2-EGFP-3Flag/BRD7 or pIRES2-EGFP and quantification. **d** Cell cycle analysis in MCF-7 and MDA-MB-231 cells transfected with pIRES2-EGFP-3Flag/BRD7 or pIRES2-EGFP and quantification. **e** Flow cytometric analysis for cell apoptosis in MCF-7 and MDA-MB-231 cells transfected with pIRES2-EGFP-3Flag/BRD7 or pIRES2-EGFP and quantification. Data are expressed as the mean ± S.D. **P < 0.01, ***P < 0.001 vs vector

### Effects of altered BRD7 expression on aerobic glycolysis

We detected the mRNA and protein expressions of BRD7 in MCF-7 and MDA-MB-231 cells transfected with BRD7 siRNAs (siRNA #1 or siRNA#2). The results show that the expression of BRD7 was significantly reduced in MCF-7 and MDA-MB-231 cells compared with the control group (Fig. 3a, b). To determine the effect of altered BRD7 expression on aerobic glycolysis in breast cancer cells, overexpression experiment of BRD7 were performed in HER2-negative MCF-7 and MDA-MB-231 cells and HER2-positive MDA-MB-453 cells. As a result, ectopic expression of BRD7 decreased lactate production, LDH activity and increased ATP production, PDH activity in breast cancer cells (Fig. 3c, e, g, supplementary 3a–c). Conversely, loss of BRD7 in MCF-7 and MDA-MB-231 cells did the opposite (Fig. 3d, f, h). Several studies have reported glycolytic inhibitors, 2-DG and oxamate, are useful in the treatment of solid tumors by attacking anaerobic cells^23^. We wondered whether BRD7 expression is correlated with the sensitivity of cells to glycolytic inhibitors. As expected, overexpression of BRD7 enhanced the inhibitory effects of these two glycolytic inhibitors on cell proliferation (Fig. 3i, j), and knockdown BRD7 presented the the opposite results in MDA-MB-231 cells (Supplementary Fig. 3d, e). Therefore, the above results demonstrate that BRD7 could reduce aerobic glycolysis and increase the sensitivity of breast cancer cells to glycolytic inhibitors.

RETRACTED

**Fig. 3:** BRD7 inhibits lactate production and LDH activity in breast cancer cells. **a** qPCR analysis of the expression of BRD7 in MCF-7 and MDA-MB-231 cells transfected with BRD7 siRNAs (siRNA #1 or siRNA#2). **b** Western blot analysis of the expression of BRD7 in MCF-7 (left) and MDA-MB-231 (right) cells transfected with BRD7 siRNAs (siRNA #1 or siRNA#2). **c** The lactate concentrations were determined in MCF-7 and MDA-MB-231 cells transfected with pIRES2-EGFP-3Flag/BRD7 or pIRES2-EGFP. **d** The lactate concentrations were determined in MCF-7 and MDA-MB-231 cells transfected with BRD7 siRNA pools (siRNA#1 and siRNA#2) or scramble siRNA (NC). **e** LDH activity was determined in MCF-7 and MDA-MB-231 cells transfected with pIRES2-EGFP-3Flag/BRD7 or pIRES2-EGFP. **f** The LDH activity was determined in MCF-7 and MDA-MB-231 cells transfected with BRD7 siRNA pools (siRNA#1 and siRNA#2) or scramble siRNA (NC). **g** ATP concentrations and PDH activity was determined in MCF-7 and MDA-MB-231 cells transfected with pIRES2-EGFP-3Flag/BRD7 or pIRES2-EGFP. **h** ATP concentrations and PDH activity were determined in MCF-7 and MDA-MB-231 cells transfected with BRD7 siRNA pools (siRNA#1 and siRNA#2) or scramble siRNA (NC). **i** MCF-7 and MDA-MB-231 cells with ectopic expression of BRD7 were treated with oxamate sodium (Oxamate) for 48 or 72 h. The cell viability was measured using an MTT assay, and the cells transfected with pIRES2-EGFP were used as a negative control. **j** MCF-7 and MDA-MB-231 cells with ectopic expression of BRD7 were treated with various concentrations of 2-DG for 48 h. The cell viability was measured using an MTT assay, and the cells transfected with pIRES2-EGFP were used as a negative control. Data are presented as the percentage of viability inhibition. *P < 0.05, **P < 0.01, ***P < 0.001

### BRD7 functions as a negative regulator of LDHA

LDHA is a key checkpoint of glycolysis that catalyzes the conversion of pyruvate to lactate^24^. We previously showed that inhibition of LDHA by inhibitors such as oxamate or siRNA can enhance the sensitivity of drug-resistant breast cancers to trastuzumab or taxol treatment^25,26^. To investigate whether dynamic expression of BRD7 could impact the expression of the key glycolysis gene LDHA, we analyzed the mRNA and protein expression of LDHA using qPCR and western blotting analysis in MCF-7, MDA-MB-231, and MDA-MB-453 cells after ectopic expression of BRD7. The results demonstrate that the mRNA and protein levels of LDHA in BRD7-overexpressed breast cancer cells were significantly lower than those in control cells (Fig. 4a, b, Supplementary Fig. 1a–c). Conversely, BRD7 silencing upregulated the expression of LDHA in MCF-7 and MDA-MB-231 cells (Supplementary Fig. 1d, e). Thus, our data clearly reveal that BRD7 negatively regulates LDHA expression at both the mRNA and protein levels in breast cancer cells.

RETRACTED

**Fig. 4:** BRD7 inhibits the expression of LDHA at the mRNA and protein level in breast cancer cells. **a** qPCR analysis of the expression of BRD7 (left) and LDHA (right) in MCF-7 and MDA-MB-231 cells transfected with pIRES2-EGFP-3Flag/BRD7 or pIRES2-EGFP. **b** Western blot analysis of the expression of BRD7 and LDHA in MCF-7 (left) and MDA-MB-231 (right) cells transfected with pIRES2-EGFP-3Flag/BRD7. **c** The dual-luciferase reporter system assay evaluated the activity of the potential LDHA  promoter in MCF-7, MDA-MB-231, and HEK293 cells. **d** The dual-luciferase reporter system assay evaluated the effect of overexpression of BRD7 on the LDHA promoter activity in MCF-7, MDA-MB-231, and HEK293 cells. **e** A schematic diagram showing the location of the LDHA potential promoter region on chromosome 11 and the locations of the PCR primers for the ChIP assay. **f** ChIP-PCR analysis of BRD7 binding of fragments of the LDHA potential promoter sequence. BIRC2 was used as a positive control. P1–P9 represent the nine fragments from the LDHA potential promoter, respectively. The error bars are presented as the mean ± S.E.M. **P < 0.01, ***P < 0.001

To further explore the mechanism of BRD7 regulating LDHA expression, we first analyzed the promoter sequence of LDHA according to the literatures reported, and found that the sequence from −1683 to 138 bp might be the potential promoter region, and thus constructed a luciferase reporter plasmid integrated with this sequence (pLuc-LDHA). We then transfected pLuc-LDHA alone or co-transfected the BRD7 expression plasmid and pLuc-LDHA into HEK293, MCF-7, and MDA-MB-231 cells. As expected, the region from −1683 to 138 bp has significant luciferase activity compared to the negative control (Fig. 4c), and upregulation of BRD7 greatly decreased the luciferase activity of the LDHA promoter (Fig. 4d). These results indicate that BRD7 negatively regulates LDHA expression through inhibiting the activity of the LDHA promoter at the transcriptional level. Then we further explored the exact region that BRD7 binds to in the LDHA promoter. The promoter sequence of LDHA was divided into nine fragments based on the DNA walking method, and each of the fragments was approximately 200–240 bp in length (Fig. 4e). The ChIP-PCR analysis showed that BRD7 could directly bind to the transcriptional regulation region of BIRC2, which was used as a positive control in this experiment^5^, but could not bind to any region of the nine fragments of this LDHA promoter (Fig. 4f), suggesting that BRD7 negatively regulates LDHA expression in an indirect manner.

RETRACTED

### BRD7 destabilizes HIF1α through the ubiquitin–proteasome pathway

To find out the candidate transcription factors that could directly regulate LDHA expression and be simultaneously regulated by BRD7, we consulted the related literature and designed series of experiments. It is interesting to find that overexpression of BRD7 can decreased HIF1α protein levels with no effect on HIF1α mRNA levels under hypoxia condition (Fig. 5a, b). Meanwhile, HIF1α has been reported to be a critical oncogenetic transcription factor that directly regulates LDHA transcription^14^. Consistent with previous results, overexpression of HIF1α could upregulate the mRNA and protein expression of LDHA in MCF-7 cells (Supplementary Fig. 4a, b). HIF1α is extremely unstable in protein level for bearing the ubiquitin–proteosome degradation in normoxic conditions. Hypoxia and CoCl_2_ were able to stabilize HIF1α protein levels and lead to its rapid accumulation^27^. In addition, BRD7 decreased LDHA expression in protein level, and restoring the expression of HIF1α in the BRD7-overexpressing cells could recover LDHA protein level (Suplementary Fig. 4c). These results suggest that BRD7 decreases LDHA expression through inactivation of the HIF1α/LDHA transcription axis.

**Fig. 5:** BRD7 destabilizes HIF1α through the ubiquitin-mediated degradation. **a** The mRNA expression of BRD7, LDHA, HIF1α, and  β-tubulin were analysised by reverse transcription-PCR (RT-PCR) under hypoxia in BRD7-overexpressing cells. **b** Western blot analysis of BRD7/Flag, HIF1α, and β-tubulin  expression in MCF-7 and MDA-MB-231 cells transfected with pIRES2-EGFP-3Flag/BRD7 under hypoxia (1%O_2_) for 24 h. **c** Western blot analysis of HIF1α and  β-tubulin expression in MCF-7 cells transfected with pIRES2-EGFP-3Flag/BRD7 and treated with CoCl2 (150 μM) and MG132 (10 μM) for the indicated periods of time (0, 4, 8, 12, 16 h) (left). Quantitative results also were shown (right). **d** MCF-7 cells transfected with pIRES2-EGFP-3Flag/BRD7 or pIRES2-EGFP for 24 h and treated with CoCl_2_ (150 μM) for 24 h. Then the cells were incubated with 50 μg/ml cycloheximide (CHX) for the indicated periods of time (0, 1, 3, 6 h) (left). Lysates were harvested from the cells and analyzed by western blotting (left panel). Quantitation of HIF1α protein levels were shown in the right pane. **e** The MCF-7 cells transfected with pIRES2-EGFP-3Flag/BRD7 and pCDNA3.1-HIF1α were under hypoxia (1% O_2_) for 24 h. Cellular co-localization of BRD7 and HIF1α in MCF-7 cells was analyzed by immunofluorescence staining with anti-BRD7 and anti-HIF1α under hypoxia (1% O_2_) for 24 h. **f** MCF-7 cells transfected with the indicated pIRES2-EGFP-3Flag/BRD7 and pCDNA3.1-HIF1α were subject to immunoprecipitation (IP) respectively with anti-Flag antibodies (upper) and anti-HIF1α (down) under hypoxia (1% O_2_) for 24 h. **g** The MCF-7 cells transfected with pIRES2-EGFP-3Flag/BRD7 and pCDNA3.1-HIF1α were under hypoxia (1%O_2_) for 24 h before collection to immunoprecipitation (IP) with anti-HIF1α antibodies

We then explored the mechanism by which BRD7 downregulates the protein levels of HIF1α. As a result, in the presence of proteasome inhibitor MG132, HIF1α protein levels were strongly blocked over time and BRD7 promote the degradation of HIF1α protein under the condition of hypoxia treated with CoCl_2_ in MCF-7 cells compared to the control (Fig. 5c). To prove that BRD7 affects HIF1α protein stability, we treated the cells with the protein synthesis inhibitor CHX, and found that the half-life of HIF1α protein was obviously shortened in BRD7-overexpressing cells (Fig. 5d). These results demonstrate that BRD7 destabilizes HIF1α protein through proteasome system. To investigate the mechanism of BRD7 destabilizing HIF1α protein, we assessed the co-localization of BRD7 and HIF1α by confocal microscopy. Interestingly, the co-localization was observed between green fluorescent protein BRD7 and red fluorescent protein HIF1α in MCF-7 cells during hypoxia (Fig. 5e). Subsequently, co-IP applied to verify protein interaction between BRD7 and HIF1α. The result showed that BRD7 and HIF1α were co-immunoprecipitated with each other (Fig. 5f). Furthermore, poly-ubiquitinated HIF1α was upregulated in the BRD7-overexpressing MCF-7 breast cancer cells (Fig. 5g), indicating that BRD7 promoted the degradation of HIF1α in a ubiquitination-dependent manner. Collectively, these results suggest that BRD7 downregulates LDHA expression through increasing HIF1α ubiquitination, which promotes the degradation of HIF1α by the proteasome.

RETRACTED

### LDHA antagonizes the effects of BRD7 on glycolysis and cell growth

As LDHA is a key enzyme that catalyzes the conversion of pyruvate to lactate, we further examined whether LDHA plays a critical role in BRD7-mediated inhibition of aerobic glycolysis. As a result, BRD7-mediated inhibitory effects on aerobic glycolysis, lactate production, and LDH activity were clearly attenuated by ecoptic expression of LDHA in BRD7-overexpressing cells. Furthermore, restoring the expression of LDHA in BRD7 knockdown cells completely recovered the effects of BRD7 silencing on glycolysis (Supplementary Fig. 5). These results suggest that LDHA is critical for BRD7-mediated inhibition of aerobic glycolysis.

Since BRD7 could significantly inhibit cell proliferation and initiate apoptosis in breast cancer cells, we further investigate the effect of LDHA on BRD7-mediated tumor suppressive roles. Intriguingly, restoring the expression of LDHA in BRD7-overexpressed breast cancer cells apparently recovered the inhibitory roles of BRD7 in regulating cell proliferation, colony formation (Fig. 6a, b), and cell cycle progression from the G1 to S phase (Fig. 6c) compared with the BRD7-overexpressed MCF-7 and MDA-MB-231 cells. Moreover, restoration of LDHA in BRD7-overexpressed breast cancer cells also reversed BRD7-induced cell apoptosis (Fig. 6d). The same result was obtained in MDA-MB-453 cells (Supplementary Fig. 2a–c). Accordingly, depletion of LDHA suppressed the effects of BRD7 silencing on cancer cell growth, cell cycle, and apoptosis (Supplementary Fig. 6). Furthermore, we also examined several key molecules related to the cell cycle and apoptosis. As expected. ectopic expression of BRD7 increased the expression of c-PARP and p21, and decreased the expression of cyclin D1 and CDK4 compared with the control group. Meanwhile, restoring the expression of LDHA at least partially recovered the expression of the above molecules related to the cell cycle and apoptosis (Fig. 7a and Supplementary Fig. 2d). In contrast, the silencing of BRD7 had the opposite effect, and restoring the expression of LDHA in BRD7 knockdown cells also recovered the expression of cell cycle and apoptosis related molecules (Fig. 7b). These data demonstrate that BRD7 functions as a tumor suppressor through an LDHA-dependent mechanism, suggesting that the tumor suppressive role of BRD7 in breast cancer cells might be associated with aerobic glycolysis.

**Fig. 6:** Overexpression of LDHA rescues the suppressive effects of BRD7 on MCF-7 and MDA-MB-231 cells. **a** MTT assay was used to determine the cell viability in MCF-7 and MDA-MB-231 cells transfected with pIRES2-EGFP-3Flag/BRD7, or co-transfected with pIRES2-EGFP-3Flag/BRD7 plus pENTER/LDHA. **b** Colony formation assay was used to determine the colony-forming ability in MCF-7 and MDA-MB-231 cells transfected with pIRES2-EGFP-3Flag/BRD7, or co-transfected with pIRES2-EGFP-3Flag/BRD7 plus pENTER/LDHA and quantification. **c** Cell cycle analysis by flow cytometry in MCF-7 and MDA-MB-231 cells transfected with pIRES2-EGFP-3Flag/BRD7, or co-transfected with pIRES2-EGFP-3Flag/BRD7 plus pENTER/LDHA and quantification. **d** Cell apoptosis analysis by flow cytometry in MCF-7 and MDA-MB-231 cells transfected with pIRES2-EGFP-3Flag/BRD7, or co-transfected with pIRES2-EGFP-3Flag/BRD7 plus pENTER/LDHA and quantification. The cells transfected with pIRES2-EGFP + pENTER were used as a control. The data are presented as the mean ± S.E.M. **P < 0.01, ***P < 0.001. All experiments were performed in triplicate

**Fig. 7:** BRD7 regulates the expression of key molecules related to the cell cycle and apoptosis and inhibits tumor growth in vivo through regulation of LDHA. **a** Western blot analysis of BRD7, LDHA, c-PARP, t-PARP, Cyclin D1, CDK4, and P21 in MCF-7 and MDA-MB-231 cells transfected with pIRES2-EGFP-3Flag/BRD7 or co-transfected with pIRES2-EGFP-3Flag/BRD7 plus pENTER/LDHA. The cells transfected with pIRES2-EGFP + pENTER were used as a control. **b** Western blot analysis for BRD7, cleaved-PARP, P21, and Cyclin D1 in MCF-7 and MDA-MB-231 cells transfected with BRD7 siRNA pools (siRNA #1 and siRNA#2), or co-transfected with BRD7 siRNA pools (siRNA #1 and siRNA#2) plus LDHA siRNA. The cells transfected with scramble control were used as a negative control (NC). **c** The cells with ectopic expression of BRD7 used for in vitro experiments were sorted by GFP-mediated flow cytometry technology to ensure the transfection efficiency. As for the recovery experiment for LDHA, the sorted cells with ectopic expression of BRD7 were further transfected with pENTER/LDHA or pENTER. Then the indicated cells were injected into nude mice. Measurement of the tumor weight across groups. **d** The tumor volume was monitored every 2 days after injection.The tumors were obtained from the mice. **e** Representative images of immunohistochemical staining for BRD7, LDHA, p21, and Cyclin D1, and the markers of proliferation and apoptosis Ki67 and c-PARP in tumor tissues, and quantification of integral optical density (IOD).The error bars are presented as the S.E.M. **P < 0.01, ***P < 0.001. All experiments were performed in triplicate

RETRACTED

### LDHA can rescue the tumor suppressive effect of BRD7 on tumor growth in vivo

Since BRD7 inhibits cell proliferation through regulation of LDHA expression in vitro, MCF-7-xenografted tumor models were performed to corroborate the above results. As a result, upregulation of BRD7 significantly suppressed the tumor growth compared with the control group, while LDHA restoration dramatically increased the tumor growth rate and weight of the xenografted tumors compared with those of the MCF-7/BRD7 group (Fig. 7c, d). We also examined the expression of BRD7, LDHA, Cyclin D1, and p21 by immunohistochemistry analysis. Consistent with the results of experiments in vitro, BRD7 overexpression increased the protein level of p21 and c-PARP and decreased the expression of Cyclin D1 and Ki67, while restoring the expression of LDHA in BRD7-overexpressing MCF-7 cells reversed the expression of the above molecules related to cell proliferation and apoptosis (Fig. 7e).

## Discussion

BRD7 was initially identified as a tumor suppressor in NPC by involved in multiple pathways such as ras/MEK/ERK, Rb/E2F, and Wnt/beta-catenin, and might be a prognostic biomarker^28,29^. Here, we demonstrated that BRD7 is downregulated in breast cancer tissues compared with normal tissues and that low expression of BRD7 is a poor prognostic factor in breast cancer. Moreover, overexpression of BRD7 in breast cancer cells exhibits a dramatic tumor suppressive effect assessed by a series of in vitro and in vivo experiments. Thus, these findings suggest that BRD7 is a novel tumor suppressor in breast cancer.

One of the key characteristics of tumor cells is deregulating cellular energetics^30^. It has been reported that aberrant expression and activity of metabolic enzymes contribute to the development and progression of cancers and that they are hallmarks of cancer. An increasing amount of evidence has confirmed that aerobic glycolysis exhibits crucial roles in tumor progression^31^. As yet, there have been no reports demonstrating the association between BRD7 and glycolysis in cancer cells. In our study, we demonstrated that ectopic expression of BRD7 reduced LDH activity and lactate production, and increased ATP production and PDH activity, while reduced expression of BRD7 did the opposite, suggesting that BRD7 is a critical negative regulator of glycolysis in breast cancer. Dysregulated metabolism, which is considered a hallmark of cancer, is frequently observed in breast cancer and is associated with tumor progression and drug resistance in cancer therapy^32^. Genetic regulators such as c-Myc and PI3k/Akt regulate metabolism as well as the ER pathway^33–35^.

In our study, we found that BRD7 overexpression could decrease LDHA expression through indirect effect on the activity of LDHA promoter at the transcriptional level validated by chromatin immunoprecipitation. Therefore, the problem to be solved is how BRD7 decreases LDHA in transcription level. LDHA is the enzyme that catalyzes the conversion of pyruvate to lactate, which is considered to be a key checkpoint of glycolysis^24^. Several transcription factors, including HIF1α, KLF4, and FOXM1, have been reported to regulate LDHA expression, which results in a shift towards the Warburg effect^36–38^. And HIF1α plays a vital role in coordinating the activities of many transcription factors and signaling molecules, which impacts tumor growth and angiogenesis^39,40^. The protein levels of HIF1α are degraded through the ubiquitination-dependent proteasomal pathway by von Hippel-Lindau (VHL)-mediated polyubiquitination and subsequent proteasomal degradation in normoxia^41,42^. In recent years, lots of reports illuminate various transcription factors take participate in polyubiquitination degradation of HIF1α^43–46^. The ER is a ligand-activated transcription factor, and its could induce cell proliferation in breast cancer cells. The ER is a ligand-activated transcription factor, and its activation could induce cell proliferation in breast cancer cells. Our results show that the expression of BRD7 is associated with that of ER in breast cancer tissues shown in Table 2, which fits with the finding that depletion of BRD7 results in loss of ERα expression in breast cancer cells^47^, while ERα signaling pathway has also been reported to directly regulate HIF1α expression^9^, appearing BRD7 could positively regulate HIF1α through activation of the ERα signaling pathway. However, BRD7 was found to function as a tumor suppressor in breast cancer whether in ER-positive breast cancer MCF-7 cells or ER-negative MDA-MB-231 and MDA-MB-453 cells, supporting that BRD7 function as tumor suppressor independent of ER but other mechanism, including the regulation of BRD7 on HIF1α. As expected, BRD7 could decrease the protein stability of HIF1α via ubiquitin-mediated proteasome pathway, and recovering the expression of HIF1α could reverse the expression of LDHA, and thus restoring the expression of LDHA could reverse the inhibition effect of BRD7 on glucose glycolysis and the tumor malignant phenotype, supporting that BRD7 inhibits the Warburg effect and tumor progression through facilitating degradation of HIF1α mediated by ubiquitin–proteasome system. Under normoxia, HIF1α is hydroxylated on prolines 402 and 564 in the oxygen-dependent degradation domain by dioxyOgenase prolyl hydroxylases, and this hydroxylated form can then interact with the VHL protein, which is part of an E3 ubiquitin ligase complex, thus resulting in HIF1α polyubiquitination and subsequent proteasomal degradation^48,49^. Therefore, whether BRD7 facilitates HIF1α degradation by promoting the function of VHL or promoting the hydroxylation of HIF1α remains to be further studied.

RETRACTED

Furthermore, our study shows that overexpression of BRD7 in breast cancer cells exhibits the tumor suppressive effects that are assessed by cell viability, cell cycle, apoptosis, and xenograft tumor model, and restoring the expression of LDHA could reverse the inhibitory effect of BRD7 on cell proliferation, apoptosis, and tumor formation in breast cancer cells both in vitro and in vivo. It has been reported that LDHA was upregulated in clinical samples of esophageal squamous cell carcinoma and that LDHA knockdown could inhibit cell growth and migration in vitro and tumorigenesis in vivo by increasing cleavage of PARP and caspase 8 and downregulating cyclin D1 and activation of AKT^50,51^. Therefore, BRD7 acts its tumor suppressive function through inhibition of LDHA expression and its downstream critical molecules or pathway.

The mechanisms that alter the bioenergetic metabolism in cancer cells are still not fully understood. However, it is generally accepted that increased glycolysis offers cancer cells an advantage to allow them to better proliferate, survive, and invade. We show that BRD7 inhibits cancer cell glycolysis and growth by targeting glycolysis-related critical molecule LDHA. The upregulation of LDHA in BRD7-overexpressing cells can promote glycolysis and cell proliferation and inhibit cell apoptosis, but the opposite result was obtained with the loss of LDHA in BRD7 knockdown cells. 2-DG, a non-metabolizable glucose analog, competitively inhibits the production of glucose 6-phosphate from glucose at the phosphoglucoisomerase level, which disrupts glycolysis and induces a state of glucoprivation. And oxamate is a structural analog of pyruvate that directly inhibits the converting process of pyruvate to lactate catalyzed by LDH, therefore, both of them inhibits cell glycolysis^52^. Thus, we further confirmed the effect of BRD7 on the glycolysis-mediated growth inhibition, and found that ectopic expression of BRD7 increased the sensitivity of breast cancer cells to 2-DG and oxamate. Therefore, our data are consistent with the notion that increased glycolysis contributes to the maintenance of cancer cell malignant phenotypes, suggesting that BRD7 plays suppressive roles in breast cancer mainly or partially through the inhibition of glycolysis.

In conclusion, we demonstrated that BRD7 inhibits both aerobic glycolysis and tumor growth by blocking HIF1α/LDHA axis in breast cancer. To our knowledge, this is the first report that BRD7 downregulates LDHA through promoting HIFα degradation under hypoxic condition in human breast cancer cells, thereby suppressing the Warburg effect and preventing tumorigenesis.

RETRACTED

## Electronic supplementary material

Supplementary figures
